# A Factorization Deep Product Neural Network for Student Physical Performance Prediction

**DOI:** 10.1155/2022/4221254

**Published:** 2022-11-19

**Authors:** Xiaoxia Jiao

**Affiliations:** Department of Physical Education Bengbu University, Bengbu 233030, China

## Abstract

As we all know, sports have great benefits for students. However, with more and more learning pressure, students' physical education has not been paid attention to by teachers and parents, so the analysis and prediction of physical education performance have become significant work. This paper proposes a new method (factorization deep product neural network) for PE course score prediction. The experimental results show that, compared with the existing performance prediction methods (LR, SVM, FM, and the DNN), the proposed method achieves the best prediction effect on the sports education dataset. Compared with the traditional optimal methods, the accuracy and AUC of DNN are both improved by 2%. In addition, there is also a significant improvement in accuracy, recall, and F1. In addition, this study found that considering two or more features at the same time has a certain influence on the prediction results of students' grades. The proposed feature combination method can learn feature combinations automatically, consider the influence of first-order features, second-order features, and high-order features in the meantime, and acquire the relationship information between each feature and performance. Compared with single-feature learning, the proposed method in this paper can enhance prediction accuracy significantly. Moreover, several dimensionality reduction methods are used in this paper, and we found that the PCA model for data processing outperformed all the benchmark models.

## 1. Background

In the information age, a large amount of data has been accumulated in all walks of life, under which there is often some useful knowledge and valuable information. At present, technologies related to machine learning and data mining are widely used in business, finance, medicine, and other fields.

With the fast development of the Internet, universities have increasingly perfected their digital campuses, and all kinds of educational data have been accumulated. However, there is often some potential knowledge and information in the massive educational data that can promote the development of education. ML data mining and other related technologies are used to provide valuable information for teachers, students, and educational researchers, so as to scientifically improve teaching methods and make comprehensive management decisions. Therefore, it is worth studying the way how better teaching efficiency and educational output are obtained from the big data of education. From the 1990s to the beginning of this century, with the fast development of the Internet, the education informatization has gradually entered the network era, and distance education and online education have attracted more and more educators' attention. The current mainstream education environment can be roughly divided into traditional classroom education and new online education, such as MOOC. Educational data mining deals with various problems in teaching, practice, and educational research through theories and technologies in multiple disciplines including pedagogy, computer science, statistics, and psychology. Currently, EDM application scenarios can be mainly divided into four categories: student performance prediction, student modeling, a recommendation system, and visualization.

## 2. Related Works

At present, education quality has become the top priority in education. Improving the quality of education is one of the unyielding determinations of educators. Now many scholars have conducted research on the prediction of students' academic performance. Early research mainly focused on collecting student learning data (such as traditional classroom teaching test scores) from the educational administration system. Students' consumption behavior data are collected from students' campus cards to predict scores. Burman used the records collected by questionnaires to classify learners into high, average, and low levels according to their academic performance based on students' psychological parameters, including personality, motivation, psychosocial background, learning strategies, learning methods, and socioeconomic status, by using a multiclassifier support vector machine [1]. A team including Sweeney used SVD, SVD-KNN, factorizers, and other recommendation system methods to predict the grades of the next semester and made a comprehensive analysis of the predicted results [2]. Sweeney proposed a method of mixed decomposer and random forest to predict students' scores by taking advantage of the course scores learned by students [3]. A team including Polyzou proposed a sparse linear and low-rank matrix decomposition model to predict future course scores based on students' historical course scores [4]. Yi et al. predicted students' scores through a multikernel support vector machine combined with an optimization algorithm, and then successfully evaluated the teaching quality [5]. AI-based methods play an increasingly important role in teaching quality evaluation [6, 7] and student performance prediction [8, 9].

Recently, with the development of the Internet and the continuous improvement of online learning platforms, the data related to MOOC students' learning has attracted more and more attention from relevant researchers. A team including Jiang used the interaction records of learners' first week on the platform and the performance data of homework to predict whether learners would eventually obtain certificates based on the logistic regression model [10]. Brinton and MChiang developed an algorithmic model relying on the decomposing machine and K-nearest neighbors (KNN) to predict whether a student answers a question correctly for the first time in a MOOC [11]. Lorenzo and Gomez-Sanchez adopted logistic regression, stochastic gradient descent, stochastic forest, and support vector machine models to predict whether the indicator, compared with the previous indicator at the end of the chapter, the three participation indicators (video, exercise, and assignment), would decline [12]. Hlosta builds a student performance prediction model based on machine learning methods (logistic regression, support vector machine, random forest, naive Bayes, and integrated learning XGBoost) in accordance with the data generated in the current course to evaluate whether students have the risk of dropping out [13]. A team including Aljohani deployed a deep long and short-term memory model based on student interaction records on online platforms (such as clickstream data) to explore student performance prediction , and the results showed that the model could predict pass/fail courses in the first 10 weeks of student interaction in a virtual learning environment with an accuracy of about 90% [14].

Compared with the application of the classical ML-based model to education such as LR [15], SVM [16], Decision Tree [17], GBDT [11], and BNs [18], the DL-based model such as RNN [19] and CNN [20] can also be used to enhance the results in the field of education.

To sum up, some achievements have been made in the study of performance prediction, but there are still some problems and shortcomings.

First, in the traditional classroom grade prediction problem, the main data information comes from some data generated during the course, such as the in-class assignment grades and unit test grades. The characteristics of the course grade prediction can be achieved until the end of the course, which leads to the late predicted results, so the method has a certain lag and the data are sparse and single, so that it cannot provide effective technical support for the teaching and management work in the early stage of the course.

Second, with a lack of other relevant course grade information, the existing online platform course grade prediction research mainly focuses on the log data of learners on the learning platform, such as the learning time on the online learning platform and the number of clicks on the learning video. In addition, in existing research, manual feature engineering is commonly used, which is highly dependent on the professional knowledge and experience of engineers, which affects the prediction accuracy of the method to a certain extent.

Third, most of the data used in the existing research on performance prediction come from the dataset constructed by researchers themselves, and the data are generally not enough. For mainstream research methods such as machine learning algorithms, there are certain requirements on the amount of data. If the data are insufficient, it is difficult to train a better model, which leads to low accuracy of prediction to a certain extent. In view of the above problems, in this paper, two kinds of different data are used to put forward different performance prediction models, so as to improve the accuracy of performance prediction.

To sum up, under the background of educational data mining, this paper carries out in-depth and systematic research on student performance prediction from the perspectives of traditional classroom teaching scenarios and MOOC online platform courses. The research focus is mainly on improving the predictability and accuracy of the method. In the following sections, the main research content of this paper is briefly introduced.

## 3. Sports Course Score Prediction Model Based on Feature Combination

### 3.1. Problem Definition

Given a student feature set F determined by the student attribution features expressed as stu de nt_attr={s_1_, s_2_,…, s_m_}, course attribution features expressed as course_attri={c_1_, c_2_,…, c_n_}, and the student learning behavior feature expressed as behavior={b_1_, b_2_,…, b_k_}. Namely, F={stu de nt_attr, course_attr, bahavior}, where *m*, n, and *k* are the number of features, respectively. For the student, his final course score was y_t_. y={0,1} is a class set divided by grades, where 0 indicates a student grade failure and 1 indicates a student grade pass. Student grade prediction aims to predict the grade category y_i_ according to the student feature F.

### 3.2. Model Framework

This chapter aims at mining and analyzing the data related to students' learning based on deep learning technology to realize the accurate prediction of students' academic performance. By so doing, timely help and guidance can be provided to students at risk of failing exams. Therefore, this chapter proposes a performance prediction model (factorization deep product neural network, FDPN) based on feature combination, course attributes, and students' learning behavior features. The model framework is shown in Figure 1. The FDPN contains 3 layers:

1. Embedding layer: narrow the dimension of the original high-dimensional features and map them to the low-dimensional feature vector.
2. Concatenate layer: this layer is composed of three parts: factorization machine, DNN, and product neural network (PNN). FM is used to express first-order and second-order features, and DNN and PNN are used to represent higher-level features.
3. Prediction layer: through splicing, the low-level and high-level features are combined to get the final features with richer information, so as to better predict students' performance.

#### 3.2.1. Embedding Layer

Because the raw data are relatively sparse, a dimensional reduction is made to obtain a low-level representation of the features. Changing the initial feature to a lower-dimensional vector representation can make the data relatively dense and reduce computational effort.  Figure 2 shows the structure of the embedding layer. Mapping the output of the embedding layer could be introduced as follows:

(1) $$\begin{array}{c} a=\left[e_{1},e_{2,}\ldots e_{p}\right]\text{.} \end{array}$$

Where a represents the embedding feature, *e*_*i*_ represents number *i* embedding feature, *p* refers to the number of embedding features, and *p* ≤ (*m*+*n*+*k*).

#### 3.2.2. Concatenate Layer

*(1) Factorization machine*. The FM, as proposed by Rendle [21], is for learning feature interactions. As shown in the formula:

(2) $$\begin{array}{c} y_{fm}=w_{0}+\overset{p}{\underset{i=2}{\sum }}w_{i}e_{i}+\overset{p}{\underset{i=1}{\sum }}\sum_{j=i+1}^{p}w_{ij}e_{i}e_{j,} \end{array}$$

where w_0_, w_i_, and w_ij_ are the weights of each feature. The factorization machine is represented by a first-order feature of logistic regression learning, and the second-order features of learning information are accumulated by the dots of vector. The last output value y_fm_ in the FM layer is transferred as input to the part of the input in the prediction layer.

DNN [22] is more capable of learning. The output of the embedding layer is the input of the first hidden layer of the DNN, and the calculation formula of the first hidden layer is shown in the following formula:

(3) $$\begin{array}{c} h_{1}=f\left(w_{o}e_{p}+b_{o}\right)\text{.} \end{array}$$

Assuming that there are *l* hidden layers, which directly output *y*_*dnn*_ to the input part of the prediction layer, the final output value of DNN is shown in the following formula:

(4) $$\begin{array}{c} y_{dnn}=f\left(w_{l-1}h_{l-1}+b_{l-1}\right)\text{,} \end{array}$$

where *f* (.) is the activation function of the hidden layer, whose activation function is the ReLU [23].

*(ii) Product neural network*. The product neural network (PNN) is a feed-forward deep neural network [24] containing the product layer. In the PNN, the input information not only contains first-order feature-related information but also second-order features. Therefore, the product layer enriches the information of the input deep neural network. Its second-order features are calculated in (5), where *p* represents the inner product of the embedding layer vectors *e*_*i*_ and *e*_*j*_.

(5) $$\begin{array}{c} p=\langle e_{i}\cdot e_{j}\rangle =\left[e_{i}^{1}e_{i}^{2}\ldots e_{i}^{p}\right]\left[\begin{array}{c} e_{j}^{1}\\ e_{j}^{2}\\ \vdots \\ e_{j}^{p} \end{array}\right]=\sum_{i=1}^{p}\sum_{j=i+1}^{p}w_{ij}e_{i}e_{j}\text{.} \end{array}$$

The input vector of the PNN is composed of the first-order feature vector output by the embedding layer and the second-order feature vector generated by the interaction of the embedding layer. The calculation is shown as follows:

(6) $$\begin{array}{c} x_{pnn}=\left[a;p\right]\text{.} \end{array}$$

The final output value *y*_*pnn*_ of the PNN is calculated, as in formula (4), which distinguishes itself from the DNN by varying the input feature vector from the embedded layer to the first hidden layer. The output values of the last hidden layer node of the PNN will be transmitted directly as input to the part node of the prediction layer input.

#### 3.2.3. Prediction Layer

The prediction layer's primary task is to combine the low- and higher-order feature representations of FM, DNN, and PNN output in the network layer and predict the grade categories of the target students. More comprehensive and accurate students' performance can be predicted by integrating the features.

In this paper, features including *y*_*fm*_,*y*_*dnn*,_ *an* *d* *y*_*pnn*_ are integrated through concatenation [25]. This process can be formalized as follows:

(7) $$\begin{array}{c} f=\left[y_{fm}{;y}_{dnn}\;;\;y_{pnn}\right]\text{,} \end{array}$$

where *f* is the final feature after integrating of *y*_*fm*_,*y*_*dnn*_ *and* *y*_*pnn*_ Finally, the feature *f* is input into the perceptron of the Sigmoid [26, 27] activation function to obtain the probability of the student course grade category.

From the above, FDPN includes three parts: FM, DNN, and PNN, and the final result is obtained from the following formula:

(8) $$\begin{array}{c} g=Sigmoid\left(f\right)\text{.} \end{array}$$

### 3.3. Loss Function

This paper employs the cross-entropy loss function and employs the L2 regularization parameter [27]. The loss function of the model is as follows:

(9) $$\begin{array}{c} loss=-\frac{1}{n}\overset{n}{\underset{i=1}{\sum }}y_{i}\log\;g+\lambda {\left\|\theta \right\|}^{2}\text{,} \end{array}$$

where *n* is the total number of training data, y_i_ is the grade category of the data, *g* is the predicted probability of the number *i* grade category of the data, and *λ*‖*θ*‖^2^ is the *L*_2_ regular term, *θ* is the set of all parameters of the model.

## 4. Experiments

### 4.1. Data Set

In this study, part of the data comes from the Open University Learning Analysis Data set (OULAD), which contains basic information, registration, and learner learning activity records from seven sport online courses from 2013 to 2014.  Figure 3 shows the learning process of using the Open University platform. First of all, the Open University opens up a course for students to apply for the course registration, and then students begin their learning. The courses of the Open University usually last for nine months, and learners are required to complete corresponding learning tasks during the learning process. Finally, learners take the final examination, and the course ends.

The description of the data set is introduced in Table 1. Numbers 1 to 54 refer to the highest degree of students who register for the course, the environment index in school learning, age, times of trying a specific module, credits of students who are currently learning,…, and times of clicking additional information before the course, such as video, tape, website, environment index of learning the module, times of clicking shared information between staff before the course, times of click PDF resources like books before the course and clicking information on the website and related activities.

According to the above descriptions, 22347×33 valid data are preprocessed.

### 4.2. Evaluation Indicators

The evaluation indexes in this paper include accuracy, precision, recall, F1, and AUC (area under the curve), which measure the model classification prediction performance.

(10) $$\begin{array}{c} Accuracy=\frac{TP+TN}{TP+TN+FP+FN}\text{,}\\ Precision=\frac{TP}{TP+FP}\text{,}\\ F1=\frac{2*Precision*Recall}{Precision+Recall}\text{.} \end{array}$$

The meanings of TP, FP, FN, and TN are shown in Table 2:

## 5. Analysis

### 5.1. Influence of Different Parameters on FDPN Model Performance

#### 5.1.1. Number of Neurons in the Hidden Layer

This model contains two deep neural networks. When a network contains multiple hidden layers and the number of neurons in each hidden layer is not the same, a lot of experimentation is required. In this paper, the same number of neurons is set in the hidden layer of the two neural networks to simplify the experiment. The experimental results are shown in Figure 4 and Table 3. Six experiments are conducted in turn to change the number of neurons. From the experimental results, it can be seen that when the number of neurons is 256, the recall rate is about 95%, the AUC is about 82%, the accuracy is about 86.6%, and the precision rate is 86.8%. The model performance is optimal because, with the increase in the number of neurons, the model can learn more feature information. However, when the neurons increase to a certain number, no more effective information can be learned by the model, and even the noise that degrades the prediction performance of the model may be generated. Therefore, in deep neural network training, too many neurons should be moderated. Model training and learning comparison are needed to select the optimal number of neurons.

#### 5.1.2. Different Activation Functions

The activation function of hidden layer neurons is related to the prediction effect about DAF. Due to the binary classification model used in this paper, the model finally predicts the output unit with the Sigmoid function, and the settings of the remaining activation functions are the same. Among ReLU, Tanh, and Sigmoid, ReLU and Tanh are better used in deep learning models, so this experiment only compares the ReLU activation function and the Tanh activation function of the hidden neuron activation function.  Table 4 introduces the experimental results. We can find that, when the activation function is ReLU, the prediction accuracy, recall rate, F1, and AUC of the FDPN model are increased by about 2%, and the prediction effect of the hidden layer neuron activation function with ReLU is better than that of the Tanh function. In particular, this chapter makes use of two feed-forward neural networks, in which the ReLU activation function performs better than the Tanh function and will be used in the last part of our study.

#### 5.1.3. The Number of Layers in the Hidden Layer

The model presented in this paper contains two feed-forward neural networks, DNN and PNN, with different numbers of hidden layers and different predictive power of the models. To simplify the experiment, the number of hidden layers in two neural networks is the same; that is, the number of hidden layers is increased from 1 to 3 layers. The experimental results are shown in Table 5. From the experimental results, it can be seen that when the hidden layer is 1 and 2, the model has a good performance, and when the hidden layer is 3, the model prediction effect is significantly reduced. As the number of layers increases, the evaluation index drops, mainly because the more layers, the more complex the structure, and the larger the calculation amount, the more likely the problem of over-fitting the model will appear. Therefore, the number of layers of the hidden layer is still set to be 1 layer in the subsequent experiments of this paper.

### 5.2. Effect of the Model Structure on the Performance

The influencing factors mainly include first-order representations and second-order representations of FM learning features and different higher-order representations of DNN and PNN learning features. In this paper, the three structures are combined for learning to predict performance. In the experiments of this section, the different feature combination structures are compared to observe the effect of the structure on the model's performance. The experimental results are shown in Table 6.

Experimental results showed that the single-structure FM, DNN, and PNN slightly performed worse, and the Deep FM, DNN + PNN, and FM + PNN of both structures that have combined feature learning are slightly better than the single structure. The FDPN model is the optimal one because it considers both first, second, and two different higher-order feature representations, during which more potentially effective information is used in performance prediction. In conclusion, the FDPN performance prediction model has a significant prediction effect and can improve prediction performance.

### 5.3. Experiment Comparison

In this paper, LR, SVM, FM, DNN, DeepFM, PNN, and other deep learning models are used as comparative models. By performing comparative experiments on the sports dataset, the results are shown in Table 7 to verify that the proposed FDPN model has the best prediction performance.

The experimental results in Table 7 show that, compared with the existing performance prediction methods (LR, SVM, FM, and the DNN), this paper achieves the best prediction effect on the sports education dataset. Compared with the optimal traditional methods, DNN accuracy and AUC are both improved by 2%. In addition, there are also significant improvements in accuracy, recall, and F1. The method based on feature combination is better than the four traditional performance prediction methods. this is mainly because the traditional performance prediction method adopts features directly as a classification feature input for model learning training and only the low or high features are taken into consideration, with the exception of the different effects of low and high feature combinations on the final performance. For the other two feature combination methods (DeepFM and PNN), this paper extracts the feature information, including first and second-order features and two different higher-order features, and thus the prediction ability of the model can be greatly improved to achieve a good prediction effect. Through the experiment, the effectiveness of the model was also confirmed. We use LDA (Latent Dirichlet Allocation) and LPP (Locality Preserving Projects) methods for combination comparison. LDA is a generation model for document topics. Make a guess about the topic distribution of the document. This model can represent all topics in the document set in the form of a probability distribution and realize topic clustering and text classification through the probability distribution of each topic. LPP is a linear manifold learning algorithm, which can preserve the local manifold structure of the original dataset and keep it in low-dimensional space. LPP is completely unsupervised; the eigenvectors of LPP are statistically correlated and not orthogonal. This means that LPP does not introduce category tags in the process of feature extraction, and category tags are of great significance for guiding feature extraction for classification problems.

Table 8 shows different performances under different dimensionality reduction methods. It can be found that the FDPN model after PCA dimensionality reduction achieves the best experimental results. In addition, we can also find that compared with the FDPN model alone, the use of the LDA method does not improve the final classification results; compared with the FDPN model alone, the LPP method improves the final classification result but is not as good as the PCA method.

## 6. Conclusion

This paper presents a new feature combination and structure model for the shortcomings of existing sports course performance prediction methods. We proposed a new method (factorization deep product neural network) for PE course score prediction. The experimental results show that, compared with the existing performance prediction methods (LR, SVM, FM, and the DNN), this paper achieves the best prediction effect on the sports education dataset. Compared with the optimal traditional methods, the DNN accuracy and AUC are both improved by 2%. In addition, there are also significant improvements in accuracy, recall, and F1. The model proposed by us provides an effective method for predicting students' performance in physical education courses.

## Figures and Tables

**Figure 1:** FDPN model framework.

**Figure 2:** Structure of the embedding layer.

**Figure 3:** Learning process.

**Figure 4:** The comparison result of neural units in the hidden layer.

**Table 1:** Data description.

Number	Features	Descriptions
1	Highest degree	The highest degree of students when enrolled in the course
2	Environmental index	The environment of the area during the course
3	Age group	Students age group
4	Times of attempts	The number of times a student tried a particular module
…	…	…
52	Shared information	Times of clicking on the course and faculties' shared information before class
53	Sources	Times of clicking on the PDF resources, such as books
54	Related information	Times of clicking on the information on the website and activities related to that information

**Table 2:** Confusion matrix.

Actual situation	Predicted results	
	Positive	Negative
Positive	TP (true and positive)	FN (false and negative)
Negative	FP (false and positive)	TN (true and negative)

**Table 3:** The comparison result of neural units in the hidden layer.

Number	Accuracy	Precision	Recall	F1	AUC
32	0.8532	0.8593	0.9395	0.8976	0.8025
64	0.8590	0.8621	0.9453	0.9018	0.8082
128	0.8619	0.8634	0.9483	0.9039	0.8111
256	**0.8668**	**0.8680**	**0.9499**	**0.9071**	**0.8179**
512	0.8607	0.8656	0.9431	0.9027	0.8124
1024	0.8578	0.8647	0.9395	0.9005	0.8099

**Table 4:** The comparison result of the activation functions.

Activation functions	Accuracy	Precision	Recall	F1	AUC
*Tanh*	0.8440	0.8610	0.9209	0.8899	0.7988
*ReLU*	**0.8668**	**0.8680**	**0.9499**	**0.9071**	**0.8179**

**Table 5:** The comparison result of the layers of the hidden layers.

Numbers of layers	Accuracy	Precision	Recall	F1	AUC
1	**0.8668**	**0.8680**	**0.9499**	**0.9071**	**0.8179**
2	0.8503	0.8639	0.9275	0.8946	0.8050
3	0.7823	0.8814	0.7882	0.8322	0.7788

**Table 6:** The result of the deep learning benchmark models.

Different structures	Accuracy	Precision	Recall	F1	AUC
FM	0.8431	0.8552	0.9281	0.8902	0.7933
DNN	0.8440	0.8554	0.9294	0.8908	0.7939
DeepFM	0.8485	0.8603	0.9297	0.8937	0.8008
PNN	0.8576	0.8646	0.9392	0.9004	0.8098
DNN + PNN	0.8614	0.8660	0.9437	0.9032	0.8131
FM + PNN	0.8625	0.8670	0.9440	0.9039	0.8147
FDPN	**0.8668**	**0.8680**	**0.9499**	**0.9071**	**0.8179**

**Table 7:** The result of the benchmark models.

Models	Accuracy	Precision	Recall	F1	AUC
LR	0.7990	0.8400	0.8728	0.8561	0.7557
SVM	0.8324	0.8464	0.9229	0.8830	0.7793
FM	0.8431	0.8552	0.9281	0.8902	0.7933
DNN	0.8440	0.8554	0.9294	0.8908	0.7939
DeepFM	0.8485	0.8603	0.9297	0.8937	0.8008
PNN	0.8576	0.8646	0.9392	0.9004	0.8098
FDPN	**0.8668**	**0.8680**	**0.9499**	**0.9071**	**0.8179**

**Table 8:** The result of the benchmark dimensionality reduction models.

Models	Accuracy	Precision	Recall	F1	AUC
LDA-FDPN	0.8616	0.8628	0.9442	0.9017	0.8130
LPP-FDPN	0.8710	0.8723	0.9545	0.9115	0.8219
PCA-FDPN	**0.8789**	**0.8802**	**0.9632**	**0.9198**	**0.8294**
FDPN	0.8668	0.8680	0.9499	0.9071	0.8179

## Data Availability

The experimental data used to support the findings of this study are available from the corresponding author upon request.
